# Interpretable Model Based on Pyramid Scene Parsing Features for Brain Tumor MRI Image Segmentation

**DOI:** 10.1155/2022/8000781

**Published:** 2022-01-31

**Authors:** Mingyang Zhao, Junchang Xin, Zhongyang Wang, Xinlei Wang, Zhiqiong Wang

**Affiliations:** ^1^College of Medicine and Biological Information Engineering, Northeastern University, Shenyang 110169, China; ^2^School of Computer Science and Engineering, Northeastern University, Shenyang 110169, China; ^3^Key Laboratory of Big Data Management and Analytics (Liaoning Province), Northeastern University, Shenyang 110169, China; ^4^Institute of Intelligent Healthcare Technology, Neusoft Corporation, Ltd., Shenyang 110179, China; ^5^Acoustics Science and Technology Laboratory, Harbin Engineering University, Harbin 150001, China

## Abstract

Due to the black box model nature of convolutional neural networks, computer-aided diagnosis methods based on depth learning are usually poorly interpretable. Therefore, the diagnosis results obtained by these unexplained methods are difficult to gain the trust of patients and doctors, which limits their application in the medical field. To solve this problem, an interpretable depth learning image segmentation framework is proposed in this paper for processing brain tumor magnetic resonance images. A gradient-based class activation mapping method is introduced into the segmentation model based on pyramid structure to visually explain it. The pyramid structure constructs global context information with features after multiple pooling layers to improve image segmentation performance. Therefore, class activation mapping is used to visualize the features concerned by each layer of pyramid structure and realize the interpretation of PSPNet. After training and testing the model on the public dataset BraTS2018, several sets of visualization results were obtained. By analyzing these visualization results, the effectiveness of pyramid structure in brain tumor segmentation task is proved, and some improvements are made to the structure of pyramid model based on the shortcomings of the model shown in the visualization results. In summary, the interpretable brain tumor image segmentation method proposed in this paper can well explain the role of pyramid structure in brain tumor image segmentation, which provides a certain idea for the application of interpretable method in brain tumor segmentation and has certain practical value for the evaluation and optimization of brain tumor segmentation model.

## 1. Introduction

The results of brain tumor image segmentation can clearly show the category, location, and volume of lesion areas [1, 2]. Therefore, introducing an automatic image segmentation model into the computer-aided diagnosis (CAD) system for brain tumor images can reduce the workload of doctors [3]. As a result, the research on brain tumor image segmentation methods has become a hotspot, so more and more brain tumor image segmentation methods [4–6] have been proposed.

Although some image segmentation frameworks [7–9] based on convolutional neural networks (CNN) have shown very high performance in various CAD systems [10–14], the complexity of these machine learning models is often greatly increased in order to improve the accuracy. Complex models represented by CNN can extract image features through multilevel abstract reasoning to deal with the very complex relationship between dependent variables and independent variables, which can achieve very high accuracy. However, this complex feature extraction method not only improves the accuracy of the model but also leads to the inability to know the relationship between the prediction results generated by the model and all the features extracted by CNN, making CNN a black box model that is difficult for human beings to understand [15]. After ResNet was proposed, the depth of CNN increased significantly from the original, making the already incomprehensible model even more inexplicable. Therefore, only result-oriented evaluation criteria such as accuracy rate and error rate can be used to evaluate the credibility of the model, which is unreliable [16].

Because CNN is a black box model, the CAD system based on CNN cannot give the diagnosis basis while giving the diagnosis results, which leads to the unreliable diagnosis results [17]. Therefore, such a diagnosis method lacking human-computer interaction is difficult to be affirmed by doctors and patients [18]. At the same time, such CAD methods may also make wrong diagnosis when the instrument is subjected to some disturbances that are difficult to be detected by human beings but will affect the diagnosis results, causing serious consequences [19]. This phenomenon seriously hinders the practical application of CNN in CAD and other fields with high reliability requirements [20].

Although the CNN model has high complexity, it is not inexplicable. Using the interpretation model can improve the transparency of the black box model and give the judgment basis of the model in a way that human beings can understand [21]. The methods for interpreting the model can be divided into ante-hoc and post-hoc [22]. Among them, the post hoc method can explain the training results of the model, which is of great significance [23].

Therefore, it is particularly important for the practical application of CNN in CAD field to explain the CNN model to improve its reliability [24–26]. With the continuous development of research in the field of deep learning, some special architectures are often embedded in the newly proposed CNN model as an improvement of the model. Taking the PSPNet used in this paper as an example, the PSP structure is used to parse the scene context in the model. However, it is difficult to verify whether such a special architecture can play a role in the corresponding tasks, and it can only be evaluated by improving the accuracy of prediction results. Although the introduced special model architecture can usually improve the accuracy, these complex structures may lead to overfitting, which makes the model achieve high accuracy on the test set, but it does not have the corresponding generalization and cannot be put into practical application. Therefore, it is necessary to verify the reasons for the improvement of accuracy and ensure the relevance between the model and the task. Therefore, the intermediate results of PSP structure in PSPNet are visualized, so that the reasoning process of CNN model can be seen to users. The GradCAM method visualizes the attention of the model to features in the way of heat map and uses it to generate intermediate results in the process of model prediction, which is suitable for analyzing the prediction process of the model. In this paper, an interpretable brain tumor image segmentation framework is proposed. In the framework, PSPNet is used to segment brain tumor images, and the visualization method based on GradCAM is used to explain the pyramid structure in PSPNet. The visualization results obtained from it prove the ability of pyramid structure to extract multiscale features. Based on the visualization results, some adjustments have been made to the pyramid structure.

The remainder of this paper is structured as follows. In Section 2, the method is described in detail, including the brain tumor image segmentation module based on PSPNet and the interpretation module based on GradCAM.  Section 3 describes the experimental process and result comparison in detail, including experiments on segmentation and experiments on interpretability. And a series of discussions are carried out on the interpretability experiments. In Section 4, a conclusion is drawn.

## 2. Methods

### 2.1. Overview

The processing method for brain tumor MRI images under this framework includes an image segmentation module using PSPNet [9] and an interpretation module using GradCAM [27]. The process is shown in Figure 1. In the image segmentation module, CNN is used to extract features from the input brain tumors MRI images. After that, global context information can be constructed from these CNN features by using the pyramid pool structure in PSPNet, which can be used to establish global scene analysis on the feature map of the last layer of CNN. Then, through the upsampling operation of convolution layer, the segmentation results of MRI images of brain tumors are obtained. At the same time, in the interpretation module, GradCAM is used to visualize the global context scene analysis information constructed in pyramid pooling structure. As a feature visualization method based on gradient information, GradCAM assigns weights to each neuron according to the gradient information flowing into the last convolution layer of CNN to extract the specific semantic information retained by each neuron. In this way, GradCAM can obtain the features concerned by CNN and display these features on the original image in the form of heat map as a visualization of CNN. By analyzing the visualization results of GradCAM and the image segmentation results of PSPNet, the interpretation of the segmentation model can be obtained.

### 2.2. Using PSPNet for Brain Tumor MRI Image Segmentation

For an input brain tumor MRI image, the process of image segmentation in PSPNet is shown in Figure 2.

Firstly, the pretrained residual network ResNet is used to extract the features of brain tumor from the image. ResNet consists of a set of residual modules, which can learn residuals to prevent gradient explosion and overfitting phenomena caused by the increasing of depth. For each residual module, setting the input of the residual module as *x* and the output of the residual module as *y*. Then, the definition of a residual block can be obtained:

(1) $$\begin{array}{c} y=F\left(x,\left\{W_{i}\right\}\right)+W_{s}x, \end{array}$$

where the function  *F*(*x*, {*W*_*i*_}) represents the learned residual mapping and *W*_*s*_ means matching *x* and *y* when the number of channels is different.

After the feature extraction of the last convolution layer in ResNet, the obtained feature map is sent to the PSP-Module. The processing of features in PSP-Module is divided into four stages, which are used to analyze the context information in the CNN features. In each stage, pooling kernels with sizes of 1 × 1, 2 × 2, 3 × 3, and 6 × 6 are used to pool the feature map. The pooling result of the feature map is used as the representation of four different scale-level subregions, and then, these feature maps need to be concatenated. However, since pooling layers of different sizes are used in each stage, the sizes of feature maps that output by each stage are also inconsistent, making it impossible to directly concatenate these feature maps. Therefore, in the PSP-Module, after the pooling layer of each stage, a 1 × 1 convolution layer is used to reduce the dimension of the output of the pooling layer, and then, four feature maps with the same size as the original feature map are obtained by interpolation. Therefore, different levels of features are concatenated to obtain the final pyramid pool features, which carry both local and global context information.

For the context information obtained by PSP-Module, three deconvolution layers are used to upsample the feature map. Finally, these feature maps are input into a 1 × 1 convolution layer to obtain the final pixel-by-pixel prediction results for brain tumors and complete the segmentation of brain tumor MRI images.

### 2.3. Using GradCAM to Interpret the Model

In order to explain the PSPNet segmentation model trained with brain tumors MRI images, the processing of visual interpretation using GradCAM is applied on it, which is shown in Figure 3. The visualization process on the PSPNet can be mainly divided into the visualization on the CNN features, the visualization on the four multiscale features, and the visualization on the context features obtained by the final concatenation.

Although the high complexity of PSPNet model usually requires a large GPU memory and takes a long time to train a high-precision model, it takes little time and computational effort to visualize the PSPNet model by GradCAM. GradCAM uses gradient to calculate the heat map during the prediction process of the model. Therefore, GradCAM does not need to modify the structure of the original model or retrain the model, so it can quickly get visual results for analysis.

#### 2.3.1. Visualization on the CNN Features

For the CNN features extracted by ResNet from brain tumors MRI images, GradCAM can be directly used to visualize them, which is shown in Figure 4. In brain tumor segmentation using PSPNet, the model will focus on the category of brain tumor, while the neurons contained in the last convolution layer in ResNet retain semantic information for identifying this category. GradCAM can be used to assign weights to each neuron in this convolution layer according to gradient information flowing into it. The semantic information in these neurons determines whether ResNet can successfully identify the category of brain tumors, and these weights represent how much influence each neuron can make on the decisions given by ResNet. In order to calculate these weights, the class of brain tumor is set as *C*, and then *y*^*c*^ is the semantic information for ResNet to judge the class as *C*. In GradCAM, the gradient information of *y*^*c*^ to feature map *A*^*k*^ is calculated by back propagation, which is *∂y*^*c*^/*∂A*^*k*^. Then, the global-average-pooling is carried out on gradient information in the width and height dimensions (indexed by *i* and *j*, respectively) of the feature map *A*^*k*^. So the weight of the kth neuron for class *C* is obtained, which is *α*_*k*_^*c*^:

(2) $$\begin{array}{c} \alpha_{k}^{c}=\overset{\text{global average pooling }}{\overbrace{\frac{1}{Z}\sum_{i}\;\sum_{j}\;}}\underset{\text{gradients via backprop }}{\underset{⏟}{\frac{\partial y^{c}}{\partial A_{ij}^{k}}}}. \end{array}$$

Next, weighted linear fusion is performed on the feature maps in all neurons with these weights. Then, ReLU is performed on the fusion results to activate the feature map which has a positive impact on the brain tumor category concerned by the ResNet model, thereby obtaining the class-discriminative localization map of Grade-CAM, which is *L*_GradCAM_^*c*^:

(3) $$\begin{array}{c} L_{\text{GradCAM}}^{c}=\text{ReLU}\underset{\text{linear combination }}{\underset{⏟}{\left(\sum_{k}\;\alpha_{k}^{c}A^{k}\right)}}. \end{array}$$

Therefore, by using gradient information to calculate, GradCAM method can realize visual interpretation of CNN features extracted from the model without modifying and retraining the PSPNet model.

#### 2.3.2. Visualization on the Four Multiscale Features

The visualization result of CNN features is only to draw a certain area on the original image with thermal map, which lacks specific and useful semantic information and is difficult to summarize into concepts that human beings can understand. Such a simple explanation result makes the model which is still a black box, which has limited significance for brain tumor segmentation. Therefore, GradCAM needs to be used to visualize the features with context semantics in PSP-Module, so that the model can be interpreted with more specific feature information. The process of visualization on the PSP-Module features using GradCAM is shown in Figure 5.

In PSP-Module, in order to extract global context information from CNN features of brain tumors extracted by ResNet, the process of extracting multiscale features is divided into four stages. Therefore, it is necessary to use GradCAM to visualize the results of CNN features in the four stages, so as to verify that each stage can extract features of different scales accordingly and contribute to the context features finally concatenated by PSP-Module. By visualizing the PSP-Features, more detailed interpretation results can be obtained from it than from the visualization of CNN features.

GradCAM itself is proposed to explain the process of extracting CNN features, so it can visualize the features extracted by ResNet in the interpretation of brain tumor segmentation However, in PSP-Module, GradCAM cannot be directly used to visualize these four multiscale features, because practical visualization results cannot be obtained through such processing. In PSP-Module, through the process of pooling and interpolation to filter the information, only the CNN features at the current scale are retained in each stage. After that, the process of concatenating the original CNN features and the CNN features at a certain scale is equivalent to weighting the original CNN features at a certain scale. This model design makes these CNN features at a certain scale show practical significance only when they are fused with the original CNN features, and it is difficult to be visualized separately. Therefore, the visualization of multiscale features is replaced by an equivalent way. In each stage, the CNN features at this scale are fused with the original CNN features, and then, the fused features are visualized by GradCAM, so that the visualization on the four multiscale features can be obtained.

#### 2.3.3. Visualization on the PSP Context Features

For the context features obtained by concatenated in PSP-Module, GradCAM is used to visualize them directly, which is similar to those described in Section 2.3.1. Combined with the features extracted from ResNet and the visualization results of multiscale features under the four stages in the pyramid structure, the visual interpretation of the multiscale feature fusion process of PSPNet can be realized.

## 3. Experiments

### 3.1. Datasets

The public brain tumor segmentation dataset BRATS2018 [28] was used in the experiment. Three segmentation targets are set in the dataset according to the type of the tumor region, including whole tumor (WT), tumor core (TC), and enhancing tumor (ET). The dataset contains 351 cases, and each case contains data collected in four modes, including T1, T2, Flair, and T1ce. Flair is used for WT and TC segmentation, and T1ce is used for ET segmentation. The data of each modality of each case is a 3D MRI image with sizes of (155, 240, and 240). The 3D brain MRI images are cut into 155 2D images, and the gray-scale value of the ground truth (GT) is used as the threshold to separate the GT of the three segmentation targets. In the experiment, PSPNet is used for brain tumor image segmentation, and dice coefficient between GT and segmentation result is taken as optimization objective and evaluation index:

(4) $$\begin{array}{c} \text{Dice}=\frac{2\left|X\cap Y\right|+\text{smooth}}{\left|X\right|+\left|Y\right|+\text{smooth}}, \end{array}$$

where smooth = 1.0, *X* is GT, and *Y* is the segmentation result.

### 3.2. Experiments on Segmentation

In order to get consistent and clear segmentation results, whole tumor lesion is chosen as the segmentation target, which is more convenient for analysis and more suitable for the visual interpretation. Additionally, in order to explain the model from multiple angles including good results and poor results and leave a certain space for the improvement ideas based on the interpretation results, the experiment uses few iterations and small batch size to limit the performance of the segmentation model in a certain extent. Therefore, in the experiment, batch size is set to 8 and epoch is set to 10. In addition, all the experiments use the learning-rate of 10^−4^ and the drop rate of 0.01. The comparison of the segmentation results is shown in Table 1.

### 3.3. Experiments on Interpretation

#### 3.3.1. Explanation on the Validity of Pyramid Structure

*(1) Visualization of Pyramid Structure*. In order to illustrate the effectiveness of pyramid structure, the input and output, as well as the intermediate results of pyramid structure, are visualized. The experimental results are shown in Figure 6, which visualizes and compares the poor and the good segmentation result, respectively. As shown in the figure, the visualization results of different scales show consistency in easily identified tumor core parts, while focusing on different regions in other details. For example, the 3 × 3 pooling in Figure 6(a) and the 6 × 6 pooling in Figure 6(b) are both focused on the bottom right region of the tumor. In contrast, other stages of the pyramid model pay less attention to this area and pay more attention to other areas. By comparing the visualization results and the label, it can be concluded that these regions are the lesions. Therefore, these stages make their contribution to the final concatenated features as shown in the PSP-Features in the figure. The experimental result interpretably proves that the pyramid structure can extract features of different scales from the input image by pooling the extracted features in multiple dimensions and then concatenate these features to obtain the final multiscale features. The output obtained by concatenated features is also very close to the label of the input image, which proves the effectiveness of pyramid structure on extracting multiscale features in an interpretable way. Therefore, introducing the pyramid structure into the model does have a positive effect on the performance improvement of the model.

*(2) Comparison between PSPNet and UNet*. Similar to multiscale feature structure of PSPNet, UNet [8] also has the ability to extract multiscale features, so the performances and visualization results of the two models are also compared in the experiment. According to the multiscale structure characteristics of UNet, a visualization method similar to PSPNet is adopted, which is interpreted based on GradCAM. The visualization results are shown in Figure 7. Through observation, it can be found that only conv_1 layer is the most similar to label in the multiscale feature extraction process of UNet, which affects the segmentation results through horizontal connection structure. Although other convolution layers can extract high-level semantic features, the features have nothing to do with both the label and output, which have no positive effect on tumor segmentation. This result proves that although UNet can extract and fuse multiscale features with the U-shape structure, the multiscale feature structure of PSPNet is much better than that of UNet in the heat map of GradCAM, and the segmentation result of PSPNet is indeed better than that of UNet.

#### 3.3.2. Analysis on the Segmentation Error

*(1) Interpretation and Analysis of Segmentation Errors*. In addition to explaining the performance of pyramid structure, it is necessary to study the reason of segmentation error in the experiment. As shown in the visualization results of PSPNet in Figure 8, the visualization result of PSP-Features is similar to GT and Output in the case of good segmentation. However, in the case of poor segmentation, the visualization result of PSP-Features is more similar to GT. It can be suspected that this phenomenon leads to the fact that most lesion areas are not accurately identified and segmented in images with poor segmentation results. The PSP-Module feature maps contain these lesion regions in a certain extent. However, the visualization results of the feature maps output by PSP-Module include these lesion regions to a certain extent, but the extracted relevant features are sparse due to reasons such as insufficient obvious features of the lesion regions, resulting in errors in the following pixel-level segmentation process. This defect of the model makes it difficult to recognize and segment these brain tumor images accurately.

In order to understand and analyze this phenomenon, this paper uses an evaluation method to further evaluate it quantitatively. Use PSNR between PSP-Features and Output, PSP-Features, and GT to measure whether the visualization result of PSP-Features is more similar to Output or GT. Therefore, it is necessary to binarize the heat map of PSP-Features. By using different thresholds to limit the range of features selected from the heat map, multiple groups of PSP-Features processed by binarization are obtained. Then, PSP-Features processed by binarization is used to calculate the PSNR value with Output and GT, respectively, and take the average value to obtain the data shown in Table 2, which is plotted as shown in Figure 9. This evaluation method makes it possible to correlate the threshold in the binarization process with the weights in CNN features to simulate the heat map that can be obtained when the weights of all features are increased in PSP-Features and quantify the effect of increasing the weights on the segmentation results.

Comparing the data in the table and the statistical chart, it can be found that when it is close to the initial weight of the features in the heat map, which means threshold = 0.45, it is more similar between PSP-Features and GT than PSP-Features and Output. However, as the threshold decreases, the weights of other features in the heat map gradually increase, and PSP-Features gradually becomes more similar to Output from being similar to GT. Especially when the threshold is reduced to 0.25, the PSNR of PSP-Features and GT reaches the highest and starts to be higher than that of PSP-Features and Output. This situation shows that at this threshold, the features of PSP-Features are the most similar to GT and more similar than Output. If the subsequent processing can be performed with the PSP-Features under this threshold, better segmentation results can be obtained. Therefore, it can be considered that PSPModule can extract the inconspicuous features of these areas and locate these focus areas to a certain extent. However, due to the defects of the model, there are problems in pixel recognition of these areas, and this defect can be improved by increasing the weight of features.

*(2) Improvement and Optimization Based on Visualization*. Since the segmentation errors in PSPNet, an idea can be applied to improve the pyramid structure to improve its performance. Because the multiscale features extracted by some stages of the pyramid structure are better in the visualization results, the weights of these scales are increased in the experiment, which makes them have more influence on the output results of pyramid structure. It can be considered that 2 × 2 and 3 × 3 are similar to GT, but the fusion process dilutes these features, resulting in darker colors and poor feature concentration in the heat map under the segmentation error in Figure 8(a). Increasing their weights can fill this deficiency and provide more appropriate scene analysis ability. However, the characteristics of 1 × 1 and 6 × 6 are less important in comparison but still need to be preserved. Therefore, in the experiment, the ratio of 1 × 1, 2 × 2, 3 × 3, and 6 × 6 was set to 1 : 2 : 2 : 1. After increasing the weight of the 2 × 2 and 3 × 3 stage in PSPNet, the dice coefficient rises to 0.5702. The visualization results are shown in Figure 10. It can be observed that increasing the weight of the scale through the concatenated features can make the feature map which is much closer to GT, thus obtaining better segmentation results. Similarly, it is not difficult to find that the color of these regions in the heat map tends to be brighten after weighting, and the segmentation result is also greatly improved. After the comparison of visualization results and the improvement of segmentation effect, it can be considered that increasing the weight of these feature scales is beneficial to improve the accuracy of brain tumor segmentation.

#### 3.3.3. Analysis on the Structure of PSPNet

*(1) The Number of Scales in Multiscale Features*. Considering the improvement of feature fusion results by increasing the weight of scales according to feature extraction ability, it is considered that the influence of changing the number of scales on feature fusion and segmentation results should also be paid attention to as another improvement idea. Therefore, in order to find a more suitable number of feature dimensions in the pyramid structure, some attempts are made to change the model by increasing or decreasing the number of scales to control the extracted features, thus seeking to improve the performance of the model. The visualization results of this experiment are shown in Figure 11. Increasing the number of scales makes the pooling scales into [1–3, 6, 8, 12], respectively. According to the visualization results, it is considered that increasing the number of scales will make the pyramid structure's ability to extract multiscale features invalid, and the features extracted by each scale tend to be consistent, resulting in a decline in model performance. However, reducing the number of scales makes the pooling scales into 2 × 2 and 3 × 3, respectively. Observing the visualization results of each scale and feature fusion in Figure 12, it can be found that reducing scales will make the pooled features of each scale scattered, unable to focus on the target tumor itself, and also make the pyramid model invalid. This problem leads to the inability to clearly locate the outline of tumor in the result of feature fusion. Therefore, the segmentation visualization results show that scale = 4 is the best number of dimensions of pyramid structure. Increasing or decreasing the number of scales on this basis will have a negative impact on the feature extraction ability of pyramid structure model.

*(2) Overfitting Problem of Pyramid Structure*. In the process of model training with 6 stages, it is inevitable that the multiscale features extracted in each scale tend to be consistent, which means that the multiscale feature structure tends to be overfitted. In order to increase the number of training iterations and apply various methods to improve the model and at the same time ensure the effectiveness of extracting multiscale features from pyramid structure, it may be necessary to introduce a penalty function based on visualization results in the training process. When the scale features extracted by pyramid structure are basically the same, it is urged to extract other neglected features to limit the overfitting degree of the model.

## 4. Conclusion

In this paper, a visualization-based interpretation method is proposed to explain the image segmentation network based on the multiscale feature model, which is used to segment MRI images of brain tumors. After training and testing the model on the public brain tumor MRI image dataset, the interpretation results prove the effectiveness of the pyramid structure, and a series of experiments are carried out based on the interpretation results to improve the performance of pyramid structure.

## Figures and Tables

**Figure 1:** The process of interpretable segmentation for brain tumors MRI image.

**Figure 2:** Using PSPNet for brain tumor MRI image segmentation.

**Figure 3:** Using GradCAM to interpret PSPNet.

**Figure 4:** Visualization on the CNN features using GradCAM.

**Figure 5:** Visualization on the PSP-Features using GradCAM.

**Figure 6:** Four groups are selected from the visualization results of PSPNet for analysis, including the ones with poor segmentation performance (a, b) and the ones with good segmentation performance (c, d). Among them, 1 × 1, 2 × 2, 3 × 3, and 6 × 6, respectively, represent the visualization of the pooling results under the four feature scales, while PSP-Features represents the fusion results of the four pooling scales in PSPNet.

**Figure 7:** Visual interpretation of multiscale features of UNet.

**Figure 8:** Comparison of PSPNet visualization results with output and label is divided into the groups with poor performance (a) and good performance (b).

**Figure 9:** Comparison of PSNR between PSP-Features and Output, PSNR between PSP-Features, and GT under binarization treatment with different thresholds.

**Figure 10:** Visual interpretation of the weighted pyramid structure.

**Figure 11:** Visualization result of increasing the number of stages in pyramid structure.

**Figure 12:** Visualization result of decreasing the number of stages in pyramid structure.

**Table 1:** The comparison of the segmentation results.

	WT	TC	ET
UNet	0.2979	0.3410	0.2812
PSPNet	0.4719	0.3763	0.2886

**Table 2:** Comparison of PSNR between PSP-Features and Output, PSNR between PSP-Features, and GT under binarization treatment with different thresholds.

Threshold	0.05	0.10	0.15	0.20	0.25	0.30	0.35	0.40	0.45
Output	12.57	14.49	15.93	17.39	18.87	20.21	21.28	21.54	21.45
GT	13.34	15.46	16.96	18.28	19.03	18.98	18.53	17.90	17.38

## Data Availability

The data used to support the findings of this study are included within the article.
